# Cross-Cultural Education and College English Speculative Reading Teaching in Multi-Modal Theoretical Environment

**DOI:** 10.1155/2022/7672692

**Published:** 2022-09-08

**Authors:** Yan Huang, Xianqing Xia

**Affiliations:** ^1^School of Foreign Languages, East China Normal University, Shanghai 200000, China; ^2^School of English, Zhejiang Yuexiu University of Foreign Languages, Shaoxing 312000, China; ^3^Shaoxing Maternity and Child Health Care Hospital, Shaoxing 312000, China

## Abstract

Due to the extensive development of globalization, the ethnic makeup of the world is becoming more and more complex, and the issue of cultural diversity has emerged as a key concern for all nations' educational systems. Cross-cultural education is an educational prescription for many western countries to deal with cultural diversity and strengthen national cohesion in order to address this issue and promote mutual respect, understanding, and communication between different groups and individuals. One of the most recent developments in global education is cross-cultural education, which has also given rise to a brand-new area of study in the field of education. The research has identified cross-cultural education as making up about 50% of all education. Numerous nations have practiced cross-cultural education, which has been promoted by UNESCO, with many issues that merit study. The traditional English teaching approach cannot meet the learning needs of today's students in light of the recent curriculum reform, and students have long engaged in passive learning. College English instructors must modify traditional teaching philosophies, adapt to contemporary developments, integrate information technology, use a variety of teaching techniques, fully pique students' interest in learning, and encourage them to take the initiative in their own education if they want to reclaim the initiative from the students in their classrooms.

## 1. Introduction

Massive multi-modal data are widely available in the age of big data. The main focus of big data research at this point, as well as the main distinction between big data and conventional data learning tasks, is how to extract the hidden great value of data through the complementary learning between modal data. College English language skills like listening, speaking, reading, writing, and translating are supported by vocabulary learning, which is the foundation of the primary stage of English language instruction. A lot of people with cross-cultural communication skills are urgently needed in this situation, so cross-cultural education has taken the top spot in English major education and teaching in colleges and universities. After graduation, English majors will be responsible for carrying out the crucial task of cross-cultural communication, so developing students' critical and inventive thinking skills is extremely important from a practical standpoint [1]. Intercultural education is particularly important. Especially, the humanity of language determines that English learners can shoulder the important task of cross-cultural communication. However, the reality of college English teaching ignores the integration of language and culture, and students' ability to recognize, analyze, explain, and create the target language culture, which is not conducive to students' mastery of cross-cultural knowledge, the development of cross-cultural communication, and the improvement of their ability to think and innovate. The expansion of human-computer interaction applications is somewhat constrained by intentional understanding based on a single modality, but the expression of a single modality can reduce user interaction load and boost interaction effectiveness in straightforward interaction scenarios. In colleges and universities, comprehensive English is a required course for English majors. It is a thorough professional basic course designed to enhance students' translation, reading, speaking, and listening skills. The majority of students' foundational vocabulary, grammatical understanding, and reading proficiency have been acquired throughout the teaching of thorough English courses. “Multi-modal discourse” teaching research has become a hot topic in the field of foreign language teaching research as a result of the ongoing development of network technology, multimedia technology [2], and corpus research.

Since China's entry into WTO, foreign exchange activities in all walks of life have increased the demand for foreign language talents, but at the same time, higher and more comprehensive requirements have been put forward for English knowledge and ability of all kinds of talents. In recent years, with the acceleration of globalization, the cooperation and competition between China and other countries have become increasingly frequent, and the exchanges between Chinese civilization and world culture have been surging. Under the background of mutual learning between Chinese and foreign civilizations, China urgently needs talents with cross-cultural ability. Synonymous vocabulary teaching also plays an important role in college English teaching. However, in fact, the actual effect of college vocabulary teaching is not good. The majority of students lose their subjective interest in learning because they perceive vocabulary instruction as tedious and tasteless. An incomplete multi-modal data fusion algorithm [3] based on deep semantic matching is proposed in order to address the issue that the existing incomplete multi-modal analysis fusion algorithms find it challenging to learn the semantics of cross-modal data sharing effectively. A unified depth model of coupled modal private depth network and incomplete modal sharing feature learning is created using the high-level semantic abstraction properties of deep learning networks. This model realizes the depth-related fusion of incomplete multi-modal data and lowers the semantic deviation of modal sharing features.

In this paper, the corresponding research methods are used to analyze and explain it. In the research of multi-modal teaching theory, the corresponding formulas and model diagrams are established to analyze them. In the related research of college English, a corresponding data map is established to analyze and explain it.

The main contributions of this paper are

1. In the article, we use the method of multi-evidence to analyze and understand.
2. In the article, the argument method is used to further explain and explain it.
3. The contribution of this paper is to use the multi-mode teaching method to further understand college English and other related contents.

The rest of this paper is arranged as follows: The second part introduces the related work to make corresponding research and ask questions. The third part studies the research and methods of multi-mode teaching and other related contents. The four parts are related to the research and analysis of college English. The fifth part summarizes the full text.

## 2. Related Work

Talents who are proficient in reading and writing trained in traditional courses can no longer meet the requirements of foreign language talents in today's society. Therefore, English communicative competence in social and cultural background, especially in cross-cultural social and cultural background, has become the main training goal of comprehensive English curriculum. In order to better understand users' intentions in different interactive situations, researchers gradually try to fuse different modal information as a means to understand complex users' intentions. Multi-modal information fusion has advanced significantly recently. With the widespread use of multimedia technology and the abundance of data description tools in the age of big data, multi-modal data are now a common occurrence. Data obtained from various fields or perspectives are referred to as multi-modal data, and each field or perspective that describes these data is referred to as a modality. The essential phase of big data analysis and mining is multi-modal data fusion. The design of fusion methods, however, is severely hindered by the multi-modal data's high-dimensional properties, modal imbalance, and modal incompleteness. In multi-modal data, modal incompleteness is the loss of some modal information for some data instances. For instance, most multi-modal text instances in multilingual text classification contain all language descriptions, whereas some text instances only contain one or a few language descriptions.

In the research, Song and Genying think that there are four levels: the first level notices some superficial cultural characteristics [4]. The second level is to be aware of some meaningful cultural features that are significantly different from the other's culture and your own. At the third level, we can understand the different cultural characteristics which are significantly different from our own culture theoretically or rationally. The fourth level is that you can put yourself in the other person's shoes and truly understand what the other person is doing. P. I. K., Bush think that it is enough to remember more words, do more reading exercises, and learn the language well, ignoring the accumulation of knowledge in other disciplines, which in turn leads to the narrow knowledge, poor critical thinking ability, and lack of creativity of English majors [5]. Aftene is of the opinion that only a natural environment is best for learning a language. A thorough English course must therefore include engaging teaching scenarios. When constructing scenes, we should not only consider the veracity, tangibility, vividness, and image of the scenes but also serve as a reminder to students to take into account relevant social and cultural differences [6]. Gui-Ling is of the opinion that intercultural education should be created for all students and citizens with the goals of fostering respect for and understanding of cultural diversity; encouraging students' integration into multiculturalism from their schools, families, and communities; achieving academic success; and enhancing international understanding. This includes teaching strategies and content, teacher preparation, interactions between schools and society, and other factors. She also advocates for strengthening regional communities. Geng proposed an intention understanding algorithm and a navigation interaction method which combined multi-modal information. Aiming at the complex user intentions in virtual interaction, an intention understanding model is constructed by using multi-modal information, which can effectively help the system guess the user's current operation intentions. On this basis, an intelligent navigation algorithm is proposed to help users conduct virtual experiments efficiently and conveniently [7]. Trnavčevič and Kralj proposed a multi-modal potential sharing feature learning method based on nonnegative matrix decomposition, which revealed the hidden relationship between each instance of multi-modal data and predefined clusters by fusing graph regularization and matrix sparseness restriction. In addition, some multi-modal shared subspace learning algorithms based on spectral embedding, undirected graph model, and Gaussian process have been proposed and achieved good results [8].

## 3. Multi-Modal Research

### 3.1. Multi-Modal Teaching Theory Research

Applying multi-modal discourse analysis theory to vocabulary teaching means that in the process of vocabulary teaching, teaching can achieve the maximum effect. By displaying the teaching content in a multi-modal way, students can be stimulated to participate in the teaching activities with various senses, thus improving the students' memory effect of words. Multi-modal discourse teaching theory specifically refers to the diversified stimulation of learners' senses through various teaching modes in teaching activities, and then on the basis of the coordinated operation of learners' senses, it can deepen their impression and understanding of what they have learned and improve their ability to use different languages to participate in communicative activities. Modality means that in the process of human cognition of external things, human beings interact with the external environment through sensory systems such as vision and hearing. In this process, human beings apply language, sound, action, and other means and language signs, forming a multi-modal discourse analysis [9, 10]. The varied use of network technology and multimedia technology in applied college English teaching has promoted significant changes in college English teaching activities to some extent in the current Internet + times context. The traditional teaching approach, which focused primarily on writing and reading, has gradually been outlawed in favor of multi-modal instruction, richer teaching methods, and activities that are more vivid and engaging in the classroom. These changes can increase students' interest in learning English and enhance the organizational impact of English instruction. This study examines the use of multimedia to display visual and auditory modes during instruction as a way for teachers to foster students' multi-modal communication skills. The impact of applying the theory of multi-modal discourse analysis to the practice of teaching foreign languages has been investigated by numerous Chinese academics. According to the experimental findings, multi-modal information input can increase students' motivation to learn foreign languages and their subjective interest in doing so [11, 12]. This enhances the impact of foreign language teaching and the level of foreign language learning. The application of the multi-modal teaching mode in college English is known as multi-modal teaching in college English, as can be seen from the analysis of the multi-modal discourse. The implementation of a multi-modal teaching approach in a college English classroom must successfully integrate the teachers, the students, the learning environment, and the instructional technology. It also needs to encourage interaction and communication between the teachers and the students while ensuring the efficacy of communication. Students should use their senses to interpret various symbol systems before internalizing them into their own knowledge. In the research, the corresponding model diagrams are established to analyze and understand them, as shown in Figures 1 and 2.

In addition, with the aid of multi-modal discourse theory, English teaching activities can integrate resources and present them in a differentiated way using sound, images, and videos to create a relevant English learning context for students, guarantee that the English teaching activities carried out can satisfy the requirements of ESP teaching in application-oriented universities, and help students finish the course. Enhancing students' English knowledge application skills and cross-cultural communication skills can serve as a strong assurance for the development of students' comprehensive English quality in application-oriented universities and also serve as a source of constructive guidance for students in order to help them reach the goal of all-round development.

With the continuous development of modern teaching technology, the teaching method has gradually changed into a compound interactive teaching mode between teachers and students. Many schools have applied multimedia equipment; created multi-modal teaching situations; effectively integrated sound, video and audio; and stimulated students' sensory systems in various aspects through multi-modal communication. The following is an analysis of the significance of multi-modal teaching mode on students' vocabulary, audio-visual, speaking, and autonomous learning [13, 14]. Under the guidance of multi-modal discourse teaching theory, in the process of reforming and innovating English teaching activities, application-oriented universities can reasonably design and optimize English multi-modal teaching, provide more professional teaching guidance to students, and ensure that the influence of English teaching on students can be displayed to the maximum extent, so that students' comprehensive English learning ability can be further enhanced. Multi-mode teaching is the improvement and development of traditional teaching mode. Therefore, under the background of information age, teachers can use network computer technology to build a stable teaching structure and teaching methods. Under the multi-modal teaching mode, college English teachers should pay attention to the effectiveness of multimedia technology application. In the process of listening teaching, teachers can find that if students only listen to the recording, it is far more difficult to understand than face-to-face communication with the speaker, which shows that the combination of vision and hearing is more conducive to information exchange and understanding. According to its research, the corresponding data tables are established to analyze it, such as Tables 1 and 2.

Multi-modal reading teaching is to use a variety of media and modes in the process of communicative teaching, so that students can form their own information after understanding, and then communicate with teachers and students in reverse. In this whole teaching process, students can not only understand the grammatical meanings of various modes but also skillfully use and select modes for information exchange in visual grammar, auditory grammar, and tactile grammar, and they can independently use the network means for creative learning in extracurricular autonomous learning. Under the guidance of multi-modal discourse teaching theory, during the process of designing teaching activities, Multi-modal teaching guidance can be adopted for the teaching of reading and writing, and students can be guided to conduct in-depth and systematic exploration of applied college English knowledge under the action of scientific teaching design, so as to help students deepen their understanding of English reading and writing knowledge, provide important assistance for the cultivation of students' comprehensive English quality, and effectively cultivate their English knowledge application ability and comprehensive communication ability.

### 3.2. Multi-Modal Algorithm Research

Stage-based fusion, feature-based fusion, and semantic-based fusion are the three broad categories into which the existing multi-modal data fusion analysis methods can be divided. Cross-modal hash retrieval involves converting data from various modalities into a Hamming space made up of compact binary codes so that it can be retrieved from the query examples of one modality. The stage-based fusion algorithm does not require a consistency constraint between modal data because different modal data are used in different stages of data mining tasks, meaning that the modal data are loosely coupled. The earliest feature-based fusion method simply concatenates all modal features in series, followed by data mining tasks like clustering and classification [15, 16], which are then finished using the combined features. A cross-retrieval method that includes at least two data types is called cross-modal retrieval. Typically, there are heterogeneous differences between different modes, meaning that the feature dimensions of various modes vary. The dimensions of the data for the same mode differ when data features are extracted, taking various extraction techniques into account. It is impossible to directly determine how similar multi-modal data are because of this heterogeneous gap. According to its research, the corresponding algorithm formulas are established, such as formulas (1)–(5).

(1) $$\begin{array}{c} k_{l}x_{1}\overset{1J}{⟶}1*1x, \end{array}$$

(2) $$\begin{array}{c} 1:x-41-\text{inf}{\left|x_{1-11}\right|}^{1}, \end{array}$$

(3) $$\begin{array}{c} \text{sin}\mathbb{C}-tr1\left|-\Gamma \right|\forall t, \end{array}$$

(4) $$\begin{array}{c} \frac{x_{v}\cdot 12^{x}/11^{7}}{x}|\Gamma_{2}^{-21c}\gamma =a_{i^{\prime }}, \end{array}$$

(5) $$\begin{array}{c} \frac{{\left|{\text{max}}^{I}71/u\right||}_{l}}{1}=1^{1},1. \end{array}$$

Because hashing technology has the characteristics of fast query speed and small storage space, cross-modal hashing has great advantages in retrieval performance. In the representation of the final data, unlike the traditional cross-modal retrieval algorithm which uses real-valued data, the cross-modal hash is represented by binary code, which involves a quantization process. The unsupervised cross-modal hashing method takes into account the intra-modal and inter-modal similarity of training data to the greatest extent in the learning process of unified binary coding and hashing function, and does not use the supervision label [17]. The probability model expresses the conditional dependence structure between random variables through graphs, and it is also a probability model. Usually, the probability graph model [18] encodes the complete distribution of multidimensional space based on the graph-based representation, where the graph can be understood as a set of independent compact or decomposed representations of a specific distribution. The supervised cross-modal hashing method can further use semantic information to learn the hash code that keeps similarity, and its performance is usually better than that of the unsupervised cross-modal hashing method. According to its research, the corresponding formulas such as (6)–(8) and (9) plus (6) are established.

(6) $$\begin{array}{c} \text{arg}\left[1^{T}\frac{,1}{1^{-}},1^{1}\right)fW^{11}t+1, \end{array}$$

(7) $$\begin{array}{c} \frac{x_{xr}}{\left\|i\text{ diag}1+\left(1^{\prime }/1\right)\right\|}, \end{array}$$

(8) $$\begin{array}{c} y_{\Pi \;\sin\;11/f∤tT_{1}}, \end{array}$$

(9) $$\begin{array}{c} F\lambda +{\left({7|}_{L}^{\pi }\right)}^{'},\text{rank}\left[\bar{I},1\right)\gamma_{1}, \end{array}$$

10) $$\begin{array}{c} \frac{1}{1/x}m-\text{atangrad},\text{i}. \end{array}$$

The main purpose of multi-modal learning is to jointly learn the potential shared information of various modal data through the complementary fusion of different feature sets, so as to improve the effectiveness of data tasks. At present, many theories and technologies have been applied to multi-modal data analysis and achieved good results. The main goal of multi-modal data aggregation is to improve the accuracy of clustering results by fusing multi-data feature sets. In the past few years, the multi-modal copolymerization problem has been widely concerned, and some effective copolymerization fusion algorithms have been proposed.

## 4. Cross-Cultural Education and Research on College English Speculative Reading

### 4.1. Cross-Cultural Education Research

Cross-cultural education includes three meanings: first, it refers to the simultaneous education of multiple cultures in an environment where multiple cultures coexist, or it refers to the education of other cultures on the basis of one culture; Second, students who have grown up in a certain cultural background go to another environment with different languages, customs, habits, values, and beliefs for education; Third, it refers to setting up a special cross-cultural environment, so that learners can receive the education of nonnative languages, customs, and values. The primary research in the area of multicultural education focuses on the theoretical framework and operational organization of multicultural education. Multicultural education has been the subject of research for more than 50 years. It has involved every aspect from the standpoint of the educational discipline, including educational theory, educational policy, curriculum and instruction, educational practice and methodology, etc. The theoretical foundation of the study can be compared to a hundred blooming flowers. Many nations around the world have faced the issue that immigrants and the culture they bring are not suitable for the lifestyle of the country of immigration since the early 20th century. Some even have significant contradictions and conflicts. English literature plays a large part in cross-cultural education [19]. First of all, from the perspective of individual's intercultural communication ability, it aims at developing intercultural communication skills and promoting individual's intercultural adaptation and intercultural communication, thus forming a very rich intercultural communication theory. According to its research, the corresponding data graphs are established to analyze it, as shown in Figures 3 and 4.

In order to successfully address the challenge of cultural diversity, cross-cultural education must first respect and recognize cultural differences, which is made possible by multiculturalism's support of ethnic minorities' cultural rights. Multiculturalism views cultural diversity as a group right and places a focus on protecting minority rights, which means that the majority society should acknowledge minority members' rights to preserve their cultural identity and give their political, economic, and cultural rights special protection. With the development of intercultural education, there are more and more researches on the basic concepts of intercultural education. Because of the language habits of various countries and the different academic backgrounds of various scholars, they have different understandings and views on the basic concepts of intercultural education. With the growth of cross-cultural education and research, it is now thought of as an interdisciplinary field of applied social science and cultural education research that focuses on the explanation, adaptation, and transformation of social groups, institutions, and individuals. Its uniqueness is to focus on the growth of socialization and education in a multicultural and globally connected society. Based on the recognition of cultural diversity, it emphasizes the dialectical relationship between ethnic culture as a whole and individual actors as well as the interaction between various cultural groups and people in daily life, with the goal of resolving disputes and realizing understanding and communication through interaction. The English affix “inter-” means to express the mutual relationship. At present, the interaction between different cultures is more and more frequent. The communication between groups or individuals with different cultural backgrounds is one of the basic characteristics of today's society, and the characteristics of the relationship between ethnic groups have also changed. Cross-cultural education is emerging to meet the challenges of this era. According to the research, the corresponding data charts are established as shown in Figures 5 and 6.

There is another connection between intercultural education and civic education in terms of attaching importance to human rights, eliminating social exclusion, and promoting the development of human resources. The continuous wave of immigrants and cultural differences in post-modern society, the transition from European nation-state to multicultural society, and the decline of integration and synchronization mechanism based on cultural community have all prompted the need to integrate multi-ethnic groups into the framework of cross-cultural civic community. The proposal of cross-cultural competence originated from the need of international political and economic exchanges. Subsequently, the research on intercultural competence is still carried out according to the practical orientation. With the deepening of people's research on intercultural situations, the constituent elements of intercultural competence are gradually expanding. Most studies on intercultural competence come from the field of intercultural communication. Because the research in this field is based on the theories of communication and philosophy, it explores and explains the characteristics of cross-cultural situations and the problems that communicators have to solve. On this basis, it forms its own cross-cultural communication theory, and then constructs the cross-cultural competence model.

### 4.2. Research on College English Speculative Reading

Speculative reading teaching is a series of teaching activities in which teachers teach students how to conduct speculative reading. It is a high-level understanding of textbook articles, including the skills of article interpretation and content evaluation. Its purpose is to help students distinguish important and unimportant information, facts and opinions. In order to fill in the information gaps and arrive at a logical conclusion, it is also necessary to infer the text's implied meaning through reasoning. The definition of speculative reading instruction is “a high-level understanding of the text, which includes the skills of interpretation and evaluation, which can enable readers to distinguish between important and unimportant information, facts and opinions, and determine the author's purpose and tone; At the same time, through reasoning, the implication is deduced, the blank part of information is filled, and a logical conclusion is drawn.” Reading in English is a psychological activity that requires readers to use their intellect and common sense in order to comprehend what they are reading. The main goals of English reading are to comprehend texts and become proficient readers. They fall under the heading of cognitive psychology and mainly discuss issues such as “what is the meaning of this word or sentence” and “what is the central idea of this paragraph or this article,” with the aim of knowing what the author is saying. The deep meaning of reading is to understand why the author said so. The purpose of cross-cultural critical reading teaching for English majors in colleges and universities is to cultivate students' cross-cultural critical thinking ability, so that they can finally achieve high-level cross-cultural communication and exchange. However, because China started late in this field, there are still many practical problems in college English teaching. To carry out cross-cultural speculative reading teaching, we must change our concepts. First, we must deeply understand the importance of cross-cultural speculative ability and carry out teaching work around this understanding; second, we should fully understand and master the connotation of cross-cultural thinking ability, and take this as the starting point and the foothold to do all kinds of teaching work well; third, we should emancipate our minds, learn and introduce advanced teaching experience at home and abroad, and provide scientific theoretical basis and guidance for future teaching work; fourthly, we should change the traditional concept of opposites in time; change the way of thinking about English culture through “colored glasses”; evaluate English culture objectively, scientifically, and dialectically; and learn from the strengths of other countries. According to its research, a corresponding data map is established for analysis, as shown in Figure 7.

The critical thinking ability is based on sufficient rationality and facts, and the cultivation of theoretical evaluation is conducive for the promotion of learning. There are many foreign schools that think about it. Speculative reading requires students to be able to infer the author's main ideas and the deep meanings of the important and difficult sentence patterns according to the specific information in the text. In today's society, there is an urgent need for compound talents who can skillfully use English for in-depth communication. This objective must be pursued by English majors who want to increase their competitiveness. We must first master the principles, practical abilities, and study techniques of the English language. Second, we must improve our capacity for cross-cultural thought and be proficient in both understanding and employing English for cross-cultural communication. The development of critical thinking skills goes hand in hand with the reading process itself. College students need to develop their analytical and problem-solving skills in English reading class in addition to building a strong foundation in language skills. The formation and accumulation of culture is a social and historical phenomenon that results from social development. Different languages have different cultures, and different cultures have different habits and characteristics. English culture has its distinctive uniqueness and nationality, which is a typical symbol of ethnic differences. The level of students' cross-cultural thinking ability is the key to the success or failure of college English teaching. Therefore, after changing the concept, we must put the cross-cultural English speculative reading teaching into practice. Teachers should recommend excellent English reading materials to students in a planned way. Especially under the condition of modern network technology, students are more willing to read articles through smart phones. Teachers can send good English articles to class groups, ask students to read them, and carry out activities after reading.

## 5. Conclusion

With the 21st century upon us, developing students' cross-cultural education and critical thinking skills has grown to be a challenging task faced by educational reform in various countries. Only by improving the development of students' critical thinking skills will English majors, in particular, be able to overcome their low standing in the discipline system and increase the employability of their graduates. According to the current situation, we must increase students' learning depth if we want to increase the effectiveness of English teaching. In order to transform students' passive learning into active exploration and discovery, we must first actively promote independent inquiry learning. Second, educators should enhance guidance while allowing students to critically and logically assess other cultures. The use of a multi-modal teaching approach when teaching college English is very effective. It not only makes the monotonous and boring environment of traditional English language instruction better, but it also combines language symbols with multi-modal symbols of nonverbal forms like video, pictures, and audio in the classroom, which motivates students to learn, leads them to actively participate in teaching activities, improves their language knowledge and communication skills as a result, and supports their overall development. By considering the subject courses and creating comprehensive courses in the school curriculum, it is possible to cultivate learners' cross-cultural aptitude. At the moment, the curriculum for school education is primarily structured around subject matter, and the development of cross-cultural competence is the main method of cross-cultural education curriculum design. The development of cross-cultural competence and the development of subject competence should support one another. A cross-cultural comprehensive curriculum is created using thematic activities and is based on the experiences of the students. Cross-cultural education has gained increasing attention from all nations as a result of the 21st century's globalization process. The practical challenge necessitates the updating and enrichment of the cross-cultural education models, methods, data, and theories, as well as increased research funding.

## Figures and Tables

**Figure 1:** Multi-modal teaching model diagram.

**Figure 2:** Simulation model diagram of multi-mode principle.

**Figure 3:** Data map of cross-cultural education (1).

**Figure 4:** Data map of cross-cultural education (2).

**Figure 5:** Cross-cultural data analysis diagram (1).

**Figure 6:** Cross-cultural data analysis diagram (2).

**Figure 7:** Analysis of speculative reading data.

**Table 1:** Multi-mode teaching data sheet.

Ydbk	Rcn	Pcns
A1	23	75
A2	74	32
A3	54	42

**Table 2:** Multi-mode teaching simulation table.

Ydbk	Rcn	Pcns
Yfs	63	53
Pang	35	78
Rcds	25	25

## Data Availability

The data used to support the findings of this study are available from the corresponding author upon request.

## References

[1] Hanifi A., Theofilis V. (2014). Modal stability theory. *Applied Mechanics Reviews: An Assessment of the World Literature in Engineering Sciences*.

[2] Zhang J., Feng W., Yuan T., Wang J., Sangaiah A. K. (2022). SCSTCF: spatial-channel selection and temporal regularized correlation filters for visual tracking. *Applied Soft Computing*.

[3] Cai W., Song Y., Wei Z. (2021). Multimodal Data Guided Spatial Feature Fusion and Grouping Strategy for E-Commerce Commodity Demand Forecasting. *Mobile Information Systems*.

[4] Song J., Genying S. U. (2015). The application of multi-modal theory in the teaching of business English reading. *Business Languages and Communication*.

[5] Bush S. R. (2010). Educating students to cross boundaries between disciplines and cultures and between theory and practice. *International Journal of Sustainability in Higher Education*.

[6] Aftene D. (2012). Cross-cultural education-A new perspective of Romanian education. *Journal of European Economy*.

[7] Geng J. (2015). The cultivation of students speculative ability in college oral English teaching. *Overseas English*.

[8] Trnavčevič A., Kralj D. (2009). Methodological issues in cross-cultural and interdisciplinary research on sustainable development. *WSEAS Transactions on Communications*.

[9] Lijun L. I. (2016). On cultivating model construction of college English teaching and thinking ability. *The Guide of Science & Education*.

[10] Chen Y., Shou-Hua H. U., Xie C. X. (2018). A probe into the teaching mode of college English speculative reading-take the new edition of college English BOOK2 UNIT1 learning, Chinese-style as an example. *Education Teaching Forum*.

[11] Xiang Z. (2014). Theoretical research on visualization of schematic interactions for the teaching of reading in English. *China Educational Technology*.

[12] Chen Z., Sun L., Zhang A. (2007). Teaching college English reading by the student-centered approach. *Higher education and academic research*.

[13] Reading S. (2008). Comprehension in college English teaching. *Journal of Wuhan Institute of Shipbuilding Technology*.

[14] Qingli L. I., University C. (2018). From a philosophical perspective: metaphor and College English Reading Teaching. *Journal of Educational Institute of Jilin Province*.

[15] Ding Y., Zhang Z., Zhao X. (2022). Multi-feature Fusion: Graph Neural Network and CNN Combining for Hyperspectral Image Classification. *Neurocomputing*.

[16] Ning X., Tian W., Yu Z., Li W., Bai X., Wang Y. (2022). HCFNN: high-order coverage function neural network for image classification. *Pattern Recognition*.

[17] Fang W. (2015). College English teaching ability training mode building. *Journal of Jiamusi Vocational Institute*.

[18] Ding Y., Zhao X., Zhang Z., Cai W., Yang N (2022). Graph sample and aggregate-attention network for hyperspectral image classification. *IEEE Geoscience and Remote Sensing Letters*.

[19] Dong L. Z. (2012). An experimental study on the web technology-based social-constructive college English extensive reading teaching mode. *Journal of Xianyang Normal University*.

